# Chemical Composition Related to Antimicrobial Activity of Moroccan *Nigella sativa* L. Extracts and Isolated Fractions

**DOI:** 10.1155/2021/8308050

**Published:** 2021-10-23

**Authors:** Salima Tiji, Yahya Rokni, Ouijdane Benayad, Nassima Laaraj, Abdeslam Asehraou, Mostafa Mimouni

**Affiliations:** ^1^Team of Electrochemistry, Laboratory of Applied Chemistry, Faculty of Sciences Oujda, University Mohammed First, Oujda, Morocco; ^2^Laboratory of Bio-Resources, Biotechnology, Ethno-Pharmacology and Health, Faculty of Sciences Oujda, University Mohammed First, Oujda, Morocco

## Abstract

**Background:**

*Nigella sativa* L. (*NS*) is an aromatic and medicinal plant commonly used in Mediterranean cuisine. Its grains contain a large amount of fixed oil and have many therapeutic virtues and medicinal properties (antioxidant, antidiabetic, antimicrobial, and anticancer).

**Aim:**

The aim of this work is to study the antimicrobial activity of *Nigella sativa* L. extracts and separated fractions on various pathogenic strains and to correlate that with its chemical composition.

**Methods:**

Extracts from Moroccan *Nigella sativa* seeds were extracted using successive organic solvents, and their hexane and acetone extracts were separated by column chromatography. The chemical composition of extracts, fractions, and essential oil was determined by GC-MS and HPLC-DAD. Extracts and fractions were evaluated for antimicrobial activity through disk diffusion against Gram-positive bacteria (*Staphylococcus aureus*, *Bacillus cereus*, and *Listeria innocua)*, Gram-negative bacteria *(Escherichia coli* and *Pseudomonas aeruginosa),* and yeast (*Candida pelliculosa)* for 1 mg/mL concentration. Bacterial strains were followed to study their behaviors over time in different concentrations. The minimum inhibitory concentration of *Nigella sativa* essential oil was determined against *Staphylococcus aureus*, *Bacillus cereus*, *Escherichia coli*, and *Candida albicans*. *Results and Conclusion*. Although hexane extract was active against both types of bacteria (Gram+ and Gram−), some of its fractions were specifically active against only one type. Fraction (SH4) had the highest activity (15 mm inhibitory diameter). Acetone extract was nonactive but surprisingly resulted in specific active fractions, and the most interesting one was (SA7) that had an inhibitory diameter of 13 mm. This antibacterial effect was related to fatty acids (linoleic and palmitic acids) in (SH4) and 17 pentatriacontene in (SA7). Moreover, the antifungal activity of hexane fractions (10–13 mm) was higher than hexane extract (8 mm), but for acetone, it was the opposite. Acetone extract had a higher activity (18 mm) than its fractions (8–12 mm), except for (SA7) (19 mm). Those inhibitions were attributed to gallic acid, cysteine, and apigenin in acetone extract and cysteine with ascorbic acid in fraction (SA7). Antifungal activity of the essential oil was more pronounced than the antibacterial one. Indeed, determined MICs in the first case were on the microgram scale (MIC = 8 *μ*g/mL, *Candida albicans*), while in the second case, they were on the milligram scale (MIC = 0.96 mg/mL for *Staphylococcus aureus*, 0.5 mg/mL for *Bacillus cereus,* and 0.68 mg/mL for *Escherichia coli*). This antifungal activity was attributed to three major compounds beta-cymene, alpha-thujene, origanene, and thymoquinone. Results of strains behavior over time at different concentrations of the fractions showed all the curves went through a maximum around 20 hours and had a delay of expression of 5 hours at the start. Taking all results into count, *Nigella sativa* L. extracts and/or derived principles could form promising antimicrobial agents for therapeutical and industrial uses.

## 1. Introduction

Commonly called black cumin, *Nigella sativa* (NS) is a yearly cool temperature resistant plant in the Ranunculaceae family. NS seeds are used in traditional medicine and as a culinary spice throughout its range from the Mediterranean basin to India. In Morocco, the plant is cultivated in coastal areas in July and traditionally used to treat asthma, diabetes, and other inflammatory diseases [1]. Indeed, research has confirmed an abundance of secondary metabolites [2]. The seeds are gaining popularity for their medicinal and dietary uses, and many cooperatives view the plant as an exploitable source of oil as the argan tree [3]. In fact, Moroccan *Nigella sativa* produces high quality oil even when compared to other variants [4]. Consequently, large-scale cultivation is being considered, despite considerable variation in yield [5].

Many studies have explored the biological properties of NS [6–8]. The plant has antibacterial effects against both Gram-positive and Gram-negative bacteria [9]. In addition, the seeds have an important activity against multidrug resistant bacterial strains [10]. NS seeds also have antifungal properties because of thymoquinone [11].

Previous studies of NS focused mostly on seed extracts or essential oils [12, 13]. The diversity of chemical compounds in the extracts makes attribution of antimicrobial activity to specific compounds difficult, especially when considering toxicity. Hepatic damage can occur with an aqueous extract [14] and metabolic changes with a lipid extract [15]. Consequently, the specific chemical(s) that imparts antimicrobial properties to NS must be separated and purified for exploitation.

In this study, we investigate the antimicrobial activity of Moroccan NS fractions separated from hexane and acetone extracts and the essential oil. The level of inhibition by the fractions was evaluated against Gram-positive and Gram-negative bacteria and fungi strains and the impact of the separation process was evaluated.

## 2. Materials and Methods

### 2.1. Plant and Material

*Nigella sativa* seeds (NS) were purchased from a local market in Oujda, Morocco. Organic analytical grade np solvents (98.9%), cycloheximide, and tetracycline were supplied by Sigma-Aldrich. Silica gel was from Fluka. Mueller–Hinton medium (BIOKAR, France) and potato dextrose (BIOKAR, France) were used for microbial cultures of bacteria and yeast, respectively. The microbial strains used as targets were *Escherichia coli*, *Pseudomonas aeruginosa*, *Staphylococcus aureus*, *Listeria innocua*, *Candida pelliculosa,* and *Candida albicans*.

### 2.2. Extractions

*Nigella sativa* (NS) seeds were cleaned and reduced by a blender into a powder of 5 *μ*m. The powder was added to warm organic solvents (50°C) with a Soxhlet apparatus and a liquid-seed ratio of 7:1. Hexane and acetone were successively used for the extraction, and organic extracts obtained were concentrated under a vacuum rotatory at 40°C and conserved at a low temperature (−4°C).

The essential oil was extracted by hydrodistillation using hexane extract produced at 50°C. Hexane extract was mixed with water and then distillated for three hours at 40°C. The essential oil was collected through Clevenger and stored at −4°C.

### 2.3. Separation of Extracts

Hexane and acetone extracts were fractioned using column chromatography. Hexane extract was separated using a silica gel column with 20% hexane/80% dichloromethane eluents. Acetone extract was separated using silica gel column chromatography and a 50% cyclohexane/50% dichloromethane eluent system [7]. The separation of both extracts was at ambient temperature and pressure.

### 2.4. Characterization Analysis

#### 2.4.1. Gas Chromatography Coupled to Mass Spectroscopy (GC-MS) Analysis

Gas chromatography (GC) analysis was performed in Shimadzu GCMS-QP2010 through GC column (30 m × 0.25 mm, 0.25 *μ*m). Helium gas was utilized as carried gas, and ionization temperature was 200°C. Time analysis for extract and fractions was 28 min and essential oil analysis time was 11 min. The compound characterization was executed based on retention time and mass fragments spectral of our samples by being compared to those of the reference standards through computer library NIST147.LIB [16].

#### 2.4.2. High Performance Liquid Chromatography Coupled to a Diode Array Detector (HPLC-DAD) Analysis

HPLC analysis was completed using Waters e2695. A C18 column (5 *μ*m, 250 × 4.6 mm) was used for analytical separation. Eluents (A: water/acetic acid (2% v/v) and B: acetonitrile pH = 2.6) were used in gradient mode. The separation was performed under a flow rate of 0.9 mL/min following Mechraoui et al.'s method [17]. The injection volume of samples was 20 *μ*l, and the column temperature was set to 25°C. The components were observed by diode array detector (DAD) at 280–365 nm. [17]. Sample chromatograms were used to compare standard referring to retention time and *λ* max. The chromatographic characterization was carried out twice and results were median.

### 2.5. Antibacterial Activity

#### 2.5.1. Disk Diffusion Test

Antibacterial activity was evaluated by an agar diffusion test, followed by the Abrigach et al.'s method [18]. Agar cultures were prepared with overnight bacterial cultures of 10^8^ cells/mL. Extracts and fractions at 10 mg/mL were aseptically positioned on sterile filter paper disks (6 mm) and on Petri plates. Papers were treated with gentamicin at 40 mg/mL as a standard antibiotic against bacteria. Dimethyl sulfoxide (DMSO) was used as the negative control. Plates with extracts and fractions were maintained at ambient temperature for prediffusion for two hours, and then the disk plates were incubated at 37°C for 24 hours [19, 20]. After incubation, inhibition diameters were measured in millimeters.

#### 2.5.2. Quantitative Test

Antibacterial activity was performed on three bacterial strains (*E*. *coli*, *P*. *aeruginosa*, and *L*. *innocua*). The extract and fractions evaluated were ((FH), (SH2), (SH3), (SA7), and (SA8)). Different concentrations from 2 to 128 *μ*g/mL were employed and the results were reported as optical density (OD) graphics.

#### 2.5.3. Microdilution Test: Determination of Antibacterial MIC in Essential Oil

The antibacterial activity of the essential oil of NS was determined when using Hayes and Markovic's microdilution method [21]. 400 *μ*L of the essential oil was diluted in 1 mL DMSO. Serial concentration (500 *μ*g/mL to 1000 *μ*g/mL) dilutions were prepared and mixed with 2% of MHB (Mueller-Hinton Broth) medium and then inoculated with overnight culture (10^7^ CFU/mL) of targets [22]. The cultures were then incubated at 37°C for 24 h. The minimum inhibitory concentration (MIC) was defined using absorbance at 625 nm, which refers to the turbidity caused by microorganism's growth. The MIC was obtained from samples showing total inhibition of bacterial growth. DMSO, used as negative control, could not inhibit bacterial strains [23].

### 2.6. Antifungal Activity

#### 2.6.1. Disk Diffusion Test

The antifungal activity of extracts and fractions of NS was determined using *Candida pelliculosa* as a target, according to the Barros et al.'s [24] method. Sterile paper disks were positioned on potato dextrose agar (PDA) plates and 1% of strain suspension. Extracts and fractions at 10 *μ*g/mL were prepared and incubated at 28°C five days. Cycloheximide 0.01% (*w*/*v*) (mg/L) was the antifungal standard and the negative control was DMSO. Fungal activity results were evaluated for five days and were expressed by diameter of inhibition halo.

#### 2.6.2. Microdilution Test: Determination of Antifungal MIC of Essential Oil

The antifungal activity of NS essential oil was performed using the Chebaibi et al.'s microdilution method [25]. Serial concentrations (1 *μ*g/mL to 32 *μ*g/mL) samples were prepared and added to the *Candida albicans* suspension and 2% MHB. Samples were incubated at 28°C for 48 hours. The MIC was determined using the concentration of completely inhibited microorganism growth.

## 3. Results

### 3.1. Extraction

*Nigella sativa* (NS) extractions were successively performed by hexane, chloroform, ethyl acetate, and acetone organic solvents using Soxhlet apparatus at 50°C. The solvents were evaporated under vacuum rotary at 40°C. Hexane extract gave a yield of 34.2% and acetone extract was represented by 2.03%. *Nigella sativa* essential oil constituted 1.12% of hexane extract and 0.28% of NS seeds.

### 3.2. Separation of Hexane and Acetone Extracts

Hexane and acetone extracts were fractioned according to our previous work [7]. Hexane extract gave eight fractions (SH (1–8)) and acetone extract specified eleven fractions (SA (1–11)). Those specified fractions were the results of successive separations of the extract tell having single compounds.

### 3.3. Gas Chromatography-Mass Spectroscopy (GC-MS) Analysis

GC-MS was performed on the hexane esterified extract, the fractions from the hexane extract, and the essential oil.

The hexane esterified extract showed the presence of linoleic acid as the most abundant component (Figure 1). Palmitic acid represented a third of the fatty composition and both oleic acid and monoacetate constituted less than 3% (Table 1).

Figure 2 shows the essential oil major constituents were *β*-cymene (37.76%), *α*-thujene (13.60%), and thymoquinone (5.69%). Other components represented less than 3%. The volatile oil was distinguished by abundant hydrocarbonic and oxygenic monoterpenes (Table 2).

The hexane fractions were identified as fatty acids. Different compounds were characterized as described in our previous study [7] based on comparing retention time and mass fragments with standard. (SH1) major compounds were 17 bromopropanoic acid (9.3%), 1-octadecanol (17.79%), linoleic acid (18.29%), heptadecanoic acid (11.02%), and 9-octadecanoic acid (28.12%). (SH2) had azelaic acid (9.44%), laural dimethyl acetal (12.14%), palmitic acid (4098.98%), linoleic acid (17.10%), and heptadecanoic acid (16.35%). Fraction (SH3) had octadecanol as one major compound (87.32%) and (SH4) had hexadecane 7.9-dimethyl (9.97%), hexadecane (10.84%), tricosanoic acid (11.17%), and 17 pentatriacontene (60.37%). The (SH5) had linoleic acid (92.54%), and (SH6) had 1-octadecanol (47.22%) and oleic acid (12.34%). (SH7) presented heptadecane 2-methyl (11.68%), 9-eicosene (16.82%), palmitic acid (18.89%), 9-tricosene (9.74%), and linoleic acid (14.08%). Finally, (SH8) had 9-eicosene (16.53%), dichloroacetic acid (16.84%), palmitic acid (24.91%), octadecanol (13.23%), and stearic acid (10.49%). Only two fractions (SH3) and (SH5) had one major compound over 87%; fractions (SH2), (SH4), and (SH6) had components around 50%. Indeed, fractions of hexane extract shared many compounds such as palmitic acid, linoleic acid, and oleic acid (Table 3).

### 3.4. HPLC-DAD

The identification of the acetone extract and its fractions revealed interesting compounds. Major compounds included polyphenol derivatives. Before the column chromatography, separation, the acetone extract contained gallic acid as the most abundant constituent. Components such as thymoquinone, apigenin, naringenin, ascorbic acid, cysteine, rutin, quercetin, and kaempferol were also found in acetone extract with different proportionalities. After the separation, the compounds were purified and were concentrated in the fractions (Table 4). (SA1) had exclusively gallic acid while (SA2) had gallic acid, thymoquinone, and apigenin. Fractions (SA3) and (SA4) had mostly catechol and naringenin, but (SA7) had cysteine and rutin while (SA11) had quercetin and histidine. Overall, acetone fractions were mostly well separated and presented one, two, or three compounds in each fraction.

### 3.5. Determination of Antibacterial Activity by Disk Diffusion Assay

The hexane extract (FH) and its fractions (SH1–9) presented a notable inhibitory effect on bacterial strains (Table 5), but visibly at lower levels than those obtained with tetracycline. Fractions (SH1) and (SH2) affected Gram-positive and -negative bacteria respectively with diameter values ranges of 8–10 mm and 10–11 mm. (SH3), (SH6), and (SH7) inhibited Gram-positive bacteria (8–12 mm), while (SH4) and (SH5) inhibited Gram-negative bacteria (12–15 mm and 9-10 mm, respectively). The antibacterial activity of (SH1), (SH2), (SH3), (SH6), (SH7), and (SH8) was moderate on both Gram-positive and Gram-negative strains and (SH4) was high against Gram-positive strains. NS hexane extract presented high activity towards *L*. *innocua* (12 mm) and medium activity towards *S*. *aureus* (10 mm) and *E*. *coli* (11 mm).

The acetone extract (FA) and its fractions (SA1) and (SA11) did not show any activity against Gram-positive or Gram-negative bacteria (Table 5). While the other acetone fractions did have antibacterial properties, they were lower than those obtained with tetracycline 1 mg/mL. (SA4), (SA8), and (SA10) had medium activity towards Gram-positive bacteria (9–12 mm), and fractions (SA5) and (SA6) had low activity against both Gram-positive and –negative bacteria (9–10 mm). (SA2) and (SA3) had high activity towards *S*. *aureus* (13 mm) and low activity towards *E*. *coli* (9-10 mm) while (SA8) and (SA10) presented a high inhibitory effect on *L*. *innocua* (12 mm). (SA7) was highly active towards all bacteria strains (12-13 mm).

### 3.6. Determination of Antibacterial Activity by Quantitative Assay

Antibacterial activity of fractions (FH), (SH1), (SH2), (SA7), and (SA8) of *Nigella sativa* (NS) were selected for their inhibitory effect previously determined and on the quantity limit. The fractions were tested for their inhibition of biomass growth of pathogenic bacteria in MH Broth, and the results obtained are reported in Figure 3. These results showed that the higher the concentration of the fraction, the greater the inhibition in biomass growth of the targets (*E*. *coli*, *P*. *aeruginosa,* and *L*. *innocua*).

Every curve was labelled at the end of its evolution. On the third step, *E*. *coli* was illustrated with the dispersion of the concentration curves (Figures 3(a), 3(c), 3(f), and 3(i)), while *P*. *aeruginosa* grouped and converged to a precise point (Figures 3(b), 3(d), 3(e), and 3(g)). *L*. *innocua* curves evolved in similar fashion (Figure 3(h)). The gap between the control and the fractions against *E*. *coli* widened over time. As time increased, the gap widened and activity increased. This traduces the positive evolution of activity on *E*. *coli* strain. For *P*. *aeruginosa*, the opposite trend was observed. All curves of both the lowest and highest activity converged to a precise point at an average time. In the case of *Listeria* strain, the activities of fractions were maintained constant for 45 minutes.

If we compare the evolution of the fractions' activities based on time, the optical density decreased when the concentrations of fractions increased for all bacterial strains. At the end of the third step (*t* = 45 min), optical density varied from two to three times for *E*. *coli*, two to five times for *P*. *aeruginosa*, and four times for *Listeria*. The antibacterial activity sequences were arranged as follows:

  (**FH**) > (**SA7**) > (**SA8**) > (**SH1**) for *Escherichia coli*
  (**SH1**) > (**FH**) > (**SA3**) > (**SA7**) > for *Pseudomonas*

### 3.7. Essential Oil Antibacterial Activity: Microdilution Test

The NS essential oil was tested on three pathogenic strains (*Staphylococcus aureus* (SA), *Bacillus cereus* (BC), and *Escherichia coli* (EC)) with concentrations from 500 to 1000 *μ*g/mL (Table 6). The minimum inhibitory concentration (MIC) values obtained were 960 *μ*g/mL for SA, 500 *μ*g/mL for BC, and 680 *μ*g/mL for EC. Those values of antibacterial activity of *Nigella sativa* essential oil were average.

### 3.8. Antifungal Activity

Hexane and acetone extracts and their fractions were tested on *Candida pelliculosa* (Table 7). The compounds presented low, medium, and high activity. Acetone extract (FA) and fraction (SA7) had high activity but not comparable to the reference cycloheximide 0.01%. The fractions (SH1), (SH2), (SH3), and (SA3) presented a high antifungal activity. For the other hexane fractions, the antifungal effects were medium or low. Hexane extract gave low activity, but generated fractions were more active. Acetone extract generated fraction (SA7) that showed the same high activity as the extract; however, the other fractions were less active than their source (FA).

### 3.9. Essential Oil Antifungal Activity: Microdilution Test

NS essential oil had a minimum fungal concentration equal to 8 *μ*g/mL against *Candida albicans* strains (Table 8). The MIC was the lowest that was found in our fungal study. In general, *Nigella sativa* had high antifungal effect that makes the essential oil a specific active antifungal.

## 4. Discussion

Solvent polarity had an impact on the extracted compounds. Successive extraction was performed in order to separate the extracted compounds based on polarity. We only used hexane and acetone extracts in this study, partly due to their polarity difference. Hexane solvent is responsible for the extraction of lipophilic components such as terpenes and sterols, and acetone extracted polar compounds such as flavonoids and polyphenols. With a yield value of 34.2%, NS seeds are high in fat. Many studies reported hexane extract was the most abundant extract from NS [26–28], while acetone extract had a yield of only 2.5% [29].

The essential oil had a low yield when it is directly extracted from NS seeds (0.18%), that is the reason why hydrodistillation was necessary for the hexane extract. Indeed, Singh et al. had a similar yield of 1.2% [30]. Volatile oil yields of 0.4% to 0.44% [31] were reported from hexane extracts by hydrodistillation and with supercritical CO_2_ method, a yield of 0.1% to 0.3% [32] based on NS seeds origin.

On the esterified hexane extract, the major components were fatty acids [32, 33], both unsaturated fatty acids such as linoleic and oleic acids and saturated fatty acids such as palmitic acid [26].

Essential oil composition depends directly on its geographical origin, climate factors, extraction method, and the temperature conditions. As a result, the composition of NS essential oil could vary from a study to another. In the literature, Burits and Bucar [31] reported alphapinene and beta. Thujene constituted 0.15%, carvacrol 8.50%, and thymoquinone 35.30%. For Wajs et al. [34], the composition was 3% carvacrol and 60% *α*-cymene and thymoquinone was less than 0.05%. The essential oil from NS Indian seeds is the most similar to those seen in this study with a composition of 36.2% *β*-cymene, 11.27% thymoquinone, 10.03% *α*-thujene, 2.12% carvacrol, and 6.3% longifolene [30]. The characterization of Iranian commercial NS essential oil had carvacrol at 2.2%, thymoquinone at 2%, *β*-cymene at 41.7%, longifolene at 3.3%, and terpinol at 1.9% [35]. The composition differences could be the result of a p-cymene transformation. In fact, even differences in the composition of essential oils harvested from the same geographical origin with the same extraction method are possible [36] because oxygen can cause transformation of p-cymene into many derivative compounds.

In hexane extract fractions, many compounds were found in multiple fractions. Repetitive acquisition of constituents is a result of not only the abundance of fatty acids but also the difficulties associated with their migration through the chromatography column. Some less common compounds in hexane extracts are reported in Table 3 such as eicosadien acid, 9.12-octadecanoic acid, and pentanone dimethyl [37, 38].

The characterization of acetone extract was in line with the chemical composition reported by Mechraoui et al. [17]. In addition, the identification of acetone extract fractions was consistent with our previous studies [7] and the fractions contained compounds with interesting biological activities [39–41].

Hexane extract and isolated linoleic acid were both more active against Gram-positive bacteria [32, 42]. Fraction (SH4) had the highest antibacterial effect on *E*. *coli* and *L*. *innocua*. Harzallah reported the inhibition zone diameter on *L*. *innocua* and *E*. *coli* were, respectively, 7 mm and 4.66 mm [43]. The antimicrobial activity of fractions (SH4) and (SH7) relied on compounds 17 pentatriacontene (50%) and hexadecane which confirmed their bioactivity [44, 45].

Acetone extract (FA) had low activity towards *Staphylococcus aureus* and *E*. *coli* [17]. However, chicks fed NS acetone extract subproducts showed high activity towards *E*. *coli* in the feces [46]. Apigenin had a low antibacterial effect [47], with thymoquinone being the active part of the fraction (SA2) [48]. (SA3) was identified as catechol, a phenolic compound with interesting antibacterial activity towards Gram-positive bacteria [49] and (SA7) activity was a result of ascorbic acid and cysteine which are well known for their antibacterial properties [50, 51]. Also, acetone fraction (SA10) was active because it contained essentially rutin that resulted in antibacterial activity towards Gram-positive and Gram-negative bacteria [52–54].

The best antibacterial activity was attributed to the fraction (SA7) towards *L*. *innocua* and fraction (SH1) towards *P*. *aeruginosa*. Hexane extract had antibacterial activity against Gram-positive bacteria [55, 56] because of thymoquinone, p-cymene, and carvacrol, all good antimicrobials [57, 58]. In many studies, the antibacterial activity was attributed to the presence of fatty acids such as oleic, linoleic, and palmitic acids in the hexane extract [59–61]. After separation, the antibacterial activity of fraction (SH1) was noticed because it contained fatty acid components such as palmitic and heptadecanoic acids [44]. Fraction (SH2) activity is almost entirely due to palmitic acid (50%), linoleic acid (17%), and heptadecanoic acid (16.35%). These compounds were reported as antimicrobials [44, 62]. The activity of acetone fraction (SA7) is explained by the presence of cysteine and ascorbic acid. In fact, ascorbic acid inhibits *E*. *coli* [50] and cysteine inhibits *L*. *innocua* and *S*. *aureus* [51, 63]. The inhibitory activity of strains by fraction (SA7) could then be caused by the intervention of one or both constituents or the result of a synergic relationship between cysteine and ascorbic acid [64].

Our essential oil MIC values for *S*. *aureus* and *E*. *coli* were similar to those obtained by Ainane et al. [65], with a MIC value of 964 *μ*g/mL towards *S*. *aureus* and a MIC equal to 676 *μ*g/mL towards *E*. *coli*. Our results for *Bacillus cereus* were similar to Landa et al. [66] (MIC = 512 *μ*g/mL) but different from *S*. *aureus* (MIC = 512 *μ*g/mL) and *E*. *coli* (MIC >1024 *μ*g/mL).

The constituents of the hexane extract are hydrophobic allowing for strong interactions with the microbial membrane. As a result, alterations to the microbial membrane increases permeability and allows high consumption of the active agent by microbial cells [67].

With palmitic and heptadecanoic acids, (SH2) and (SH3) were more active than hexane extract that contains linoleic acid at 80% [62]. Machraoui et al. reported modest activity by acetone extract against *C*. *albicans* [17]. (SA2) had medium activity and contained mostly apigenin. In fact, apigenin inhibited *A*. *tenuissima* [68] which was also active through the membrane perturbation and biofilm reduction which changes *Candida* physiology [69, 70].

(SA3) caused high antifungal activity. Fungal strains are sensitive to catechol; in consequence, its antifungal activity was elevated [49, 71]. Moreover, (SA7) was the most active fraction that even exceeded the acetone extract. (SA7) contained cysteine which changes the morphology of fungal colonies by creating a structural modification that generates nuclear degradation [72, 73].

The chemical mechanism for the essential oil is difficult to explain due to its complexity. It is possible that every single component has its own mechanism of action. The most abundant compounds describe the essential oil efficacy. For example, terpenes and hydrocarbons have an inhibitory effect on bacteria strains. In fact, the lipophilic propriety of skeletal hydrocarbons and hydrophilic properties of alcohol, aldehydes, and ketones have a positive impact on antimicrobial activity [74, 75].

Thymoquinone and carvacrol in the essential oil had minimal antimicrobial activity [58, 65]. Hydrocarbons such as lilac aldehyde D in NS essential oil had high antimicrobial activity likely because conjugated aldehyde groups with double carbon-carbon bonds are highly electronegative. Suggesting that increasing electronegativity would increase antimicrobial activity [76, 77].

The presence of thymol in essential oil could show a medium activity against bacterial strains [78]. Terpenes such as *α*-pinene, *β*-pinene, and *γ*-terpinene also present high antibacterial activity towards Gram-positive bacteria and medium activity towards Gram-negative bacteria [30, 79, 80].

## 5. Conclusion

Column chromatography was used to separate hexane and acetone extracts into their purified fractions. Characterization based on GC-MS and HPLC-DAD showed the nature of the extracts and fractions and exposed links between antimicrobial activity and chemical composition.

Hexane and acetone extracts and their fractions had antibacterial and antifungal activities. Most fractions were more active against Gram-positive than Gram-negative bacteria. However, the (SH4) was active towards Gram-negative bacterial strains, and (SA7) had the highest antifungal activity.

The microdilution method was proceeded on NS essential oil for the determination of antibacterial and antifungal activities through quantification by MIC. Our results show that antifungal activity is more important than antibacterial activity.

Antimicrobial activity was a consequence of separated compounds as witnessed by comparing activity before and after separation. This may be a result of a unique isolated compound in the fraction or several compounds that react simultaneously or synergistically, meaning two compounds would individually have low activities, but when combined within the same fraction, their activity would increase. In summary, *Nigella sativa* L. extracts and fractions are interesting antimicrobials that could be exploitable in therapy and industry.

The next step is to test the active antimicrobial fractions against “sensitive” foods to determine if *Nigella sativa* can be used for food preservation.

## Figures and Tables

**Figure 1:** GC chromatogram of esterified hexane extract.

**Figure 2:** GC chromatogram of NS essential oil.

**Figure 3:** The biomass growth variation of target bacterial strains in the presence of hexane and acetone fractions.

**Table 1:** Hexane extract identification by GC-MS.

Peak	Compound	RT (min)	Area (%)
1	Oleic acid	9.93	2.74
2	Monoacetate, 1,2,3-propanetriol	11.31	2.40
3	Palmitic acid	22.58	30.33
4	Linoleic acid	24.33	64.52

RT, retention time; area, percentage obtained by electronic integration measurement using a mass detector RT trace. RT, retention time.

**Table 2:** NS essential oil characterization by GC-MS.

Peak	Compound	RT (min)	Concentration
1	Alpha-Thujene, origanene, or 3-thujene	5.00	13.60
2	Alpha-Pinene	5.13	2.20
3	Beta-Pinene	5.84	2.18
4	1,2,4-Trimethylbenzene or pseudocumene, Psi-cumene	6.10	1.30
5	Beta-Cymene	6.60	37.76
6	Gamma-Terpinene	7.15	0.69
7	Lilac aldehyde	7.79	0.55
8	2-Cyclohexen-1-ol, 2-methyl-5-(1-methylethyl)-, (1S-cis)	8.17	2.19
9	Thymoquinone	10.23	5.69

**Table 3:** Fractions of hexane extract identified by GC-MS.

Fraction	Peak number	Compound	RT (min)	Area (%)
(SH1)	1	2.4-Decadienal	15.11	4.95
	2	Lauric acid	18.68	1.87
	3	Palmitic acid	22.61	8.64
	4	17 bromopropanoic acid	23.26	9.3
	5	1-Octadecanol	23.58	17.79
	6	Linoleic acid	24.36	18.29
	7	Heptadecanoic acid	24.64	11.02
	8	9-Octadecanoic acid (Z), 2-butoxyethyl ester	25.79	28.12

(SH2)	1	8-Hydroxyoctanoic acid	16.23	2.61
	2	Methyl azelaaldehydate	16.77	2.60
	3	Azelaic acid	18.26	9.44
	4	Laural dimethyl acetal	18.89	12.14
	5	Palmitic acid	22.62	40.98
	6	Linoleic acid	24.37	17.10
	7	8-Octadecenoic acid	24.43	1.25
	8	Heptadecanoic acid	24.62	16.35

(SH3)	1	2.4-Decadienal	15.24	1.70
	2	Palmitic acid, methyl ester	22.60	5.65
	3	1-Octadecanol	23.84	87.32
	4	Oleic acid, methyl ester	24.34	5.31

(SH4)	1	7,9-Dimethylhexadecane	15.17	9.97
	2	Hexadecane	18.13	10.84
	3	Tricosanoic acid	22.58	11.17
	4	17 pentatriacontene	24.59	60.37
	5	Lignocerol	24.79	7.62

(SH5)	1	2.6.11.15-Tetramethyl hexadecane	17.55	0.29
	2	9-Eicosene (E)	18.78	1.79
	3	Palmitic acid, methyl ester	22.60	2.65
	4	(Z)-9-tricosene	23.28	2.70
	5	Linoleic acid	24.05	92.54

(SH6)	1	Eicosane	18.13	2.19
	2	Dichloroacetic acid, heptadecyl ester	18.77	4.08
	3	9-Tricosene	21.14	5.12
	4	Palmitic acid, methyl ester	22.60	4.09
	5	l-(+)-Ascorbic acid 2.6-dihexadecanoate	23.03	14.37
	6	9-Tricosene	23.28	6.60
	7	1-Octadecanol	23.91	47.22
	8	Oleic acid	24.81	12.34
	9	9-Hexacosene	25.24	3.95

(SH7)	1	2.3-Dimethylhexadecane	15.18	6.11
	2	8-Methylheptadecane	15.18	3.71
	3	2,6,11,15-Tetramethylhexadecan-	17.55	8.44
	4	Pentanoic acid, 5-hydroxy-,2,4-di-t-butylphenyl esters	17.83	3.87
	5	2-Methylheptadecane-	18.13	11.68
	6	9-eicosene (E)	18.78	16.82
	7	Dichloroacetic acid, heptadecyl ester	21.15	6.42
	8	Palmitic acid, methyl ester	22.60	18.89
	9	9-Tricosene. (Z)-	23.28	9.74
	10	Linoleic acid	24.35	14.08

(SH8)	1	2.4-Decadienal	15.16	3.82
	2	9-Eicosene. (E)-	18.77	16.53
	3	Dichloroacetic acid, heptadecyl ester	21.14	16.84
	4	Palmitic acid, methyl ester	22.60	24.91
	5	1-Octadecanol	23.58	13.23
	6	Oleic acid, methyl ester	24.39	5.57
	7	Stearic acid, methyl ester	24.62	10.49
	8	9-Hexacosene	25.23	8.59

RT, retention time; area, percentage obtained by electronic integration measurement using a mass detector RT trace.

**Table 4:** Acetone extract and its fractions identification by HPLC-DAD.

Sample	RT (min)	Area (%)	Compound
Extract (FA)	2.92	23.50	Gallic acid
	2.97	2.03	Ascorbic acid
	3.74	4.85	ND
	3.80	3.65	ND
	5.40	3.82	Thymoquinone
	19.22	4.95	Rutin
	22.28	8.45	Naringenin
	27.74	8.42	Quercetin
	32.54	2.03	Kaempferol
	42.42	13.20	Cysteine
	42.50	3.73	ND
	42.60	13.27	Apigenin
	42.73	8.05	ND

Fraction (SA1)	2.92	98.9	Gallic acid

Fraction (SA2)	2.92	25.8	Gallic acid
	5.40	12.3	Thymoquinone
	42.60	73.5	Apigenin

Fraction (SA3)	2.92	5.36	Gallic acid
	39.92	79.83	Catechol

Fraction (SA4)	22.28	88.7	Naringenin

Fraction (SA6)	3.74	10.74	ND
	42.73	86.72	

Fraction (SA7)	2.97	13.9	Ascorbic acid
	42.42	82.17	Cysteine

Fraction (SA8)	3.80	25.21	ND
	42.50	72.01	

Fraction (SA11)	19.22	4.80	Rutin
	27.74	7.65	Quercetin
	42.24	12.3	L-Histidine

ND, none determined; RT, retention time; area, percentage obtained by electronic integration measurement using a mass detector RT trace.

**Table 5:** Antibacterial activity of hexane ((FH) and (SH (1–9)) and acetone ((FA and SA (1–11)) fractions obtained from *N. sativa* seeds^∗^.

	Gram−		Gram+	
Fractions of hexane extract	*E*. *coli*	*P*. *aeruginosa*	*L*. *innocua*	*S*. *aureus*

(FH)	11	ND	12	10
(SH1)	8	10	11	ND
(SH2)	8	ND	11	10
(SH3)	ND	ND	8	10
(SH4)	15	ND	12	9
(SH5)	10	9	ND	ND
(SH6)	ND	ND	12	8
(SH7)	ND	ND	8	9
(SH8)	9	ND	ND	11
DMSO (1 mg/mL)	—	—	—	—
Tetracycline (1 mg/mL)	30	30	30	30

	Gram −		Gram+	
Fractions of acetone extract	*E*. *coli*	*P*. *aeruginosa*	*L*. *innocua*	*S*. *aureus*

(FA)	ND	ND	ND	ND
(SA1)	ND	ND	ND	ND
(SA2)	10	ND	ND	13
(SA3)	9	ND	ND	13
(SA4)	ND	ND	10	9
(SA5)	ND	9	10	10
(SA6)	10	ND	ND	9
(SA7)	10	13	12	11
(SA8)	ND	ND	12	10
(SA10)	ND	ND	12	ND
(SA11)	ND	ND	ND	ND
Tetracycline (1 mg/mL)	30	30	30	30
DMSO (1 mg/mL)	—	—	—	—

^*∗*^Values are in mm (inhibition diameter); ND, not detected; DMSO, dimethyl sulfoxide.

**Table 6:** Determination of essential oil MIC towards antibacterial strains.

	1000 *μ*g/mL	970 *μ*g/mL	960 *μ*g/mL	950 *μ*g/ml	700 *μ*g/mL	680 *μ*g/mL	500 *μ*g/mL	Control
SA	−	−	−	+	+	+	+	+
BC	−	−	−	−	−	−	−	+
EC	−		−	−	−	−	+	+

SA, *Staphylococcus aureus*; BC, *Bacillus cereus*; EC, *Escherichia coli*.

**Table 7:** Inhibition diameters (mm) of hexane and acetone fractions obtained against *Candida pelliculosa*.

Fractions from hexane extract samples	*Candida pelliculosa*

Hexane extract (FH)	8
(SH1)	13
(SH2)	12
(SH3)	12
(SH4)	10
(SH5)	8
(SH6)	10
(SH7)	10
(SH8)	11
DMSO	ND
Cycloheximide 0.01%	24

Fractions from acetone extract samples	*Candida pelliculosa*

Acetone extract (FA)	18
(SA1)	10
(SA2)	11
(SA3)	12
(SA4)	10.9
(SA5)	11
(SA6)	8
(SA7)	19
(SA8)	8
(SA10)	9
(SA11)	8
Cycloheximide 0.01%	24
DMSO	ND

ND, none determined.

**Table 8:** Determination of essential oil MIC towards antifungal strain.

Concentration (*μ*g/mL)	32	16	8	4	2	1	Control
*Candida albicans*	−	−	−	+	+	+	+

## Data Availability

All data used to support the finding of this study are available online and from the corresponding author upon request.

## Abbreviations

(FH): Hexane extract
(FA): Acetone extract
(SH (1–8)): Hexane extract separated fractions
(SA (1–11)): Acetone extract separated fractions
GC-MS: Gas chromatography-mass spectroscopy
HPLC-DAD: High performance liquid chromatography coupled with diode array detector
MIC: Minimal inhibition concentration.
